# Another reason for the counterintuitive effects of thank-you gifts on charitable giving

**DOI:** 10.3389/fpsyg.2022.908556

**Published:** 2022-07-29

**Authors:** Zhou Fang, Yong Bian

**Affiliations:** ^1^Department of Economic Sciences, Claremont Graduate University, Claremont, CA, United States; ^2^Department of Economics and Statistics, California State University, Los Angeles, Los Angeles, CA, United States; ^3^Collaborative Innovation Center of Statistical Data Engineering Technology and Application, Zhejiang Gongshang University, Hangzhou, China; ^4^International Business School, Zhejiang Gongshang University, Hangzhou, China

**Keywords:** thank-you gift, waste, donation, charitable giving, altruism

## Abstract

Current studies on the effect of thank-you gifts on charitable giving are primarily based on the conclusion of a milestone paper, “The counterintuitive effects of thank-you gifts on charitable giving” which argued that thank-you gifts are mainly driven by lower feelings of altruism. This article argues that the question design in “The counterintuitive effects of thank-you gifts on charitable giving” may lead to a biased conclusion. This article added an extra treatment group to the original study and found that the authors neglected the critical impact of participants’ inference about the usage of the money.

## Introduction

The effect of thank-you gifts is a severe concern in charity research, and most of the studies are based on the conclusion of the research article “The counterintuitive effects of thank-you gifts on charitable giving.” In their research, they argued that although people believe that thank-you gifts would raise charitable donations, the outcome is the opposite, as offering a gift reduces feelings of altruism (Newman and Shen, 2012).

Their study raised discussions in academia and the charity industry. Major social media such as Forbes, reported their result (FORBES, 2012), and follow-up studies were conducted right after the paper was published (Andrews et al., 2014; Kulow and Kramer, 2016). Ten years later, as today, the paper is still a milestone that researchers would refer to when they study altruism and gift in a donation. For example, Huang et al. (2021) followed their study to further investigate laypeople’s belief of the influence of thank-you gifts on charitable giving, which confirmed that laypeople believe thank-you gifts would raise charitable donations and one mediation of the effect is anticipated positive emotion; another study found that thank you gifts increase (decrease) the weight that donors place on self-interested (prosocial) motives, leading to changes in donation patterns as the gift may activate mindsets or norms that emphasize self-interested motives instead of more prosocial, other-regarding motives (Chao and Fisher, 2022).

While altruism certainly plays an important role in the charitable donation reductions, the authors argue that one possibility which was not considered influential in Newman and Shen’s paper (2012, p. 6) may also be a reason. In their paper, they stated that in a follow-up study, participants were asked to estimate “what percentage of donations does this charity devote to overhead costs?” to test whether participants may have inferred that the part of the donation was used to pay for the thank-you gifts themselves. The authors believe that the overhead cost is a biased estimator for “paying for gifts” for two reasons: first, gift costs can be only a small portion of the overhead costs, so offering a gift does not significantly change the participants’ estimations of the costs; second, rather than a quantitative issue, the matter can be qualitative that the gifts give a sign of “using the donation on something against my purpose.”

To determine whether such beliefs change the amount of donations, the authors first replicated the third experiment of Newman and Shen’s (2012) study and added a third treatment group to the original design. The remainder of the paper is organized as follows. Section “Experiment design” introduces the experiment design. Section “Results” presents the results. Section “Discussion and conclusion” discusses and concludes.

## Experiment design

The authors fully replicated the third experiment of Newman and Shen’s (2012) study and added a third group that is identical to the treatment group except being showed an additional statement, “The tote bags are provided by a local business for free; we do not use donations to purchase thank-you gifts,” under the picture of the tote bag (coded treatment 2 thereafter). Below are the descriptions of the experiment from Newman and Shen’s paper which the authors followed as instructions.

*“In this study, participants were asked to donate to the Save-the-Children foundation. In exchange for participating in the study, participants were entered into a lottery for a $95 gift certificate to an online retailer. They were asked how much of those winnings they would be willing to donate to the charity. At the end of the study, lottery winners were randomly selected, and the $95 was divided between the participant and the charity, as specified by the participant. Between-subjects we manipulated whether the donation request was accompanied by the offer of a thank-you gift (a tote bag bearing the Save-the-Children logo) or not (no-gift control). In cases where winning participants were assigned to the gift condition, they were provided with the tote bag along with the remaining value of the gift certificate. Following the donation, participants in both conditions were asked to rate the charity in terms of effectiveness (1* = *not at all effective, 9* = *very effective) and how wealthy (1* = *not at all wealthy, 9* = *very wealthy) they perceived the charity to be.”*

Three hundred California residents were recruited on a data collection platform, Prolific^1^, and completed our experiment on Qualtrics. Respondents were recruited from the same state to maintain the consistency of purchasing powers. The average age of the responders is 33.54 (min = 18, max = 82). 205 of them are female, 86 are male, and the rest defined themself as non-binary or third gender.

The participants were told that they would answer a survey about donations on Qualtrics, which will take 1–2 min on the Prolific recruitment page. The compensation for completing the survey was 0.3 US dollars, at the hourly rate of 9.00 US dollars for 2 min. Informed consents are obtained from all participants.

## Results

The authors first published our main results in Table 1; both the donation rates and amount are higher compared to Newman and Shen’s (2012) study, but the overall pattern of results is similar in the first two groups.

**TABLE 1:** Summary statistics of the donation questions.

Condition	Count	% Donate	Mean	Mean (d)	Med	SD	Effective	Wealthy
**No-gift (control)**	100	87	28.76	33.06	25	25.65	6.00	5.81
**Gift (treatment)**	100	76	24.01	31.59	15	25.74	5.49	5.84
**Gift. S (treatment 2)**	100	89	27.93	31.38	20	25.42	5.81	5.87

The fifth column, mean (d), calculated the average amount of actual donations (excluding 0 s).

First, with a *p*-value of 0.38 in ANOVA (as shown in Table 2), we cannot reject the means of all conditions are equal. However, if our assumptions hold, there should be a significant difference between the control group and the treatment group, but not necessarily between the control group and the second treatment group.

**TABLE 2:** ANOVA results: Means comparison between the three groups (all).

Model	DF	Sum of squares	Mean	*F*-Ratio	Prob. level	Reject equal means? (α = 0.05)
**Between**	2	1287.26	643.63	0.98	0.38	No
**Within (error)**	297	194661.7	655.42			
**Adjusted total**	299	195949				
**Total**	300					

Therefore, the authors next conducted the hypothesis tests between each of the three two-group combinations. The results of the one-sided two-sample *T*-tests are presented as following: the control group, the participants who were simply asked for a donation, donated more than the first treatment group who were offered the tote bag as a thank-you gift (*p* = 0.048, mean.c = 28.76, Sd-c = 25.65, mean.t1 = 24.01, Sd.t1 = 25.74); the difference become insignificant when compared to the second treatment group for whom the statement is given (*p* = 0.205, mean.c = 28.76, Sd.c = 25.65, mean.t2 = 27.93, Sd.t2 = 25.42); however, the difference between the control groups is only weakly significant (*p* = 0.070, mean.t1 = 24.01, Sd.t1 = 25.74, mean.t2 = 27.93, Sd.t2 = 25.42).

Similar cases apply to the medians according to the Wilcoxon signed-rank test; the median in the control group and the second treatment group are significantly larger than in the first treatment group (median.c = 25, median.t1 = 15, median.t2 = 20, *p* = 0.0245 and 0.0249, respectively). Still, there is no significant difference between the medians of the control group and the second treatment group (median.c = 25, median.t2 = 20, *p* = 0.228). Similar to the results of Newman and Shen’s (2012) study, ratings of the charity’s efficacy did not differ across conditions, nor did perceptions of the charity’s wealth (*p* > 0.1 for both *F*-tests).

The authors next tried to compare the difference in donations from the people who actually chose to donate (excluding the 0 s). We still cannot reject the equal mean hypothesis in ANOVA (*p* = 0.89, see details in Table 3), and all the *T*-test results are no longer significant (mean.c = 33.06, mean.t1 = 31.59, mean.t2 = 31.38; Sd.c = 24.77, Sd.t1 = 25.13, Sd.t2 = 24.84, *p* = 0.35, 0.48, and 0.68, respectively). These results mean that among the people who chose to donate, using thank-you gifts and statements is not making a big difference, which means the decrease in the average donation is probably caused by the lower donation rate of the first control group.

**TABLE 3:** ANOVA results: Means comparison between the three groups (donators only).

Model	DF	Sum of squares	Mean	*F*-Ratio	Prob. level	Reject equal means? (α = 0.05)
**Between**	2	143.78	71.89	0.12	0.89	No
**Within (error)**	249	154456.1	620.31			
**Adjusted total**	251	154599.9				
**Total**	252					

Therefore, the authors conducted the same tests for the dummy variable of whether the responders chose to donate. Both the participants in the control and second treatment groups are more willing to donate (mean.c = 87, mean.t1 = 76, mean.t2 = 89; Sd.c = 0.34, Sd.t1 = 0.43, Sd.t2 = 0.31) compared to the first treatment group (*p* = 0.01 and 0.02, respectively), but not for the control and second treatment group (*p* = 0.67).

## Discussion and conclusion

We replicated Newman and Shen’s (2012) study with an extra treatment as we disagree with the one of the conclusions of the paper. Our experiment showed that much of the deduction comes from the hypothesis that “participants may have inferred that the part of the donation was used to pay for the thank-you gifts themselves,” which was rejected by Newman and Shen’s (2012) study. We believe this finding would contribute to current literature about using thank-you gifts in charity fundraising.

Additionally, our finding also contributed to another stream of important research that the donors’ willingness to disregard overhead costs when someone else pays for those costs. In other words, overhead is not a problem as long as “my” donation is not used for those purposes. It was found that if participants were told the administration and other fundraising fees would be covered by a startup grant, twice as many people were willing to make donations (Gneezy et al., 2014). However, unlike other overhead costs such as administration fees, the thank-you gifts may be special. In another study, overhead aversion is still found even if other people pay for the overhead cost in fundraising (Charles et al., 2020). But in our study, the donation rate even increased (although not significant) after the statement of a “free” thank-you gift. This finding is exciting and important as if the thank-you gift does not trigger people’s overhead aversion when a third party is paying for it, it would still be beneficial to the charities if people are carrying tote bags with their logos around even if the thank-you gift does not significantly raise the donations directly.

In the end, although the authors made an argument against Newman and Shen’s (2012) study, that does not mean the authors are against the conclusion that altruism plays an important role in charity fundraising. The authors’ purpose of the study is to state that altruism and overhead aversion are both important when a thank you gift is being considered for fundraising and to find a better way to use the thank-you gifts.

## Data availability statement

The datasets presented in this study can be found in online repositories. The names of the repository/repositories and accession number(s) can be found below: https://figshare.com/articles/dataset/TYG2/20391420.

## Ethics statement

Ethical review and approval was not required for the study on human participants in accordance with the local legislation and institutional requirements. The patients/participants provided their written informed consent to participate in this study.

## Author contributions

YB collected the data. ZF completed the rest. Both authors contributed to the article and approved the submitted version.

## Footnotes

1
https://www.prolific.co

## References

[B1] AndrewsM.LuoX. M.FangZ.AsparaJ. (2014). Cause marketing effectiveness and the moderating role of price discounts. *J. Market.* 78 120–142. 10.1509/jm.14.0003 11670861

[B2] ChaoM.FisherG. (2022). Self-interested giving: the relationship between conditional gifts, charitable donations, and donor self-interestedness. *Manag. Sci.* 68 4537–4567. 10.1287/mnsc.2021.4039 19642375

[B3] CharlesC.SloanM. F.SchubertP. (2020). If someone else pays for overhead, do donors still care? *Am. Rev. Public Adm.* 50 415–427. 10.1177/0275074020913989

[B4] FORBES (2012). *Charities: Don’t Thank Your Donors with a Gift.* Available online at: https://www.forbes.com/sites/rogerdooley/2012/08/08/donor-gifts/?sh=3e48d2a210c6 (accessed February 26, 2022).

[B5] GneezyU.KeenanE. A.GneezyA. (2014). Avoiding overhead aversion in charity. *Science* 346 632–635. 10.1126/science.1253932 25359974

[B6] HuangH. Q.ZhangY. Z.LvJ. Y.JiangT.ZhangX.ChenX. H. (2021). Laypeople’s belief of the influence of thank-you gifts on charitable giving. *Soc. Psychol.* 52 331–342. 10.1027/1864-9335/a000461

[B7] KulowK.KramerT. (2016). In pursuit of good karma: when charitable appeals to do right go wrong. *J. Consum. Res.* 43 334–353. 10.1093/jcr/ucw018

[B8] NewmanG. E.ShenY. J. (2012). The counterintuitive effects of thank-you gifts on charitable giving. *J. Econ. Psychol.* 33 973–983. 10.1016/j.joep.2012.05.002

